# Analysis of Sepsis Markers and Pathogenesis Based on Gene Differential Expression and Protein Interaction Network

**DOI:** 10.1155/2022/6878495

**Published:** 2022-02-12

**Authors:** Jifang Liang, Weidong Wu, Xiuzhe Wang, Wenjing Wu, Shuxian Chen, Meini Jiang

**Affiliations:** ^1^Department of Critical Medicine, Shanxi Bethune Hospital (Tongji Shanxi Hospital of Shanxi Academy of Medical Sciences), The Third Hospital of Shanxi Medical University, 030031 Taiyuan, Shanxi, China; ^2^Department of Critical Medicine, Tongji Hospital Affiliated to Tongji Medical College of Huazhong University of Science and Technology, 430030 Wuhan, Hubei, China

## Abstract

**Objective:**

The purpose of the present study is to screen the hub genes associated with sepsis, comprehensively understand the occurrence and progress mechanism of sepsis, and provide new targets for clinical diagnosis and treatment of sepsis.

**Methods:**

The microarray data of GSE9692 and GSE95233 were downloaded from the Gene Expression Omnibus (GEO) database. The dataset GSE9692 contained 29 children with sepsis and 16 healthy children, while the dataset GSE95233 included 102 septic subjects and 22 healthy volunteers. Differentially expressed genes (DEGs) were screened by GEO2R online analysis. The DAVID database was applied to conduct functional enrichment analysis of the DEGs. The STRING database was adopted to acquire protein-protein interaction (PPI) networks.

**Results:**

We identified 286 DEGs (217 upregulated DEGs and 69 downregulated DEGs) in the dataset GSE9692 and 357 DEGs (236 upregulated DEGs and 121 downregulated DEGs) in the dataset GSE95233. After the intersection of DEGs of the two datasets, a total of 98 co-DEGs were obtained. DEGs associated with sepsis were involved in inflammatory responses such as T cell activation, leukocyte cell-cell adhesion, leukocyte-mediated immunity, cytokine production, immune effector process, lymphocyte-mediated immunity, defense response to fungus, and lymphocyte-mediated immunity. Kyoto Encyclopedia of Genes and Genomes (KEGG) pathway enrichment analysis suggested that sepsis was connected to bacterial and viral infections. Through PPI network analysis, we screened the most important hub genes, including ITK, CD247, MMP9, CD3D, MMP8, KLRK1, and GZMK.

**Conclusions:**

In conclusion, the present study revealed an unbalanced immune response at the transcriptome level of sepsis and identified genes for potential biomarkers of sepsis, such as ITK, CD247, MMP9, CD3D, MMP8, KLRK1, and GZMK.

## 1. Introduction

Sepsis is a systemic inflammatory reaction mainly caused by pathogen infection, which is often characterized by high fever, leukocytosis, and headache [1]. Sepsis can lead to multiple organ dysfunction syndrome (MODS) and circulatory failure in critical condition, which is a common acute and severe disease in clinic. The incidence rate and mortality rate of sepsis are very high. 30 million people worldwide are infected with sepsis every year, in which 8 million people are dead [2]. However, the number of morbidity and mortality has been underestimated in countries with backward development and poor economy. Therefore, sepsis has caused serious physical injury and economic pressure to human beings.

The basic reason for the poor treatment effect of sepsis is that the pathogenesis of sepsis is not clear, and there are few indicators for clinical diagnosis and prognosis of sepsis. In order to reduce the mortality of patients and improve the quality of life of patients with sepsis, relevant research has been widely carried out, but little progress has been made. With the development and application of gene chip technology, thousands of differential genes have been found. Screening the genes that play a key role in disease among many different genes has become a key research goal. Bioinformatics analysis based on gene expression profile may screen hub genes and regulatory pathways, which plays an important role in early diagnosis of sepsis and establishment of early warning mechanism.

In the research of life science, bioinformatics uses computer technology as a tool to store, retrieve, analyze, and visualize biological information. It has been widely applied to identify hub genes of diseases at the molecular level. Many bioinformatics studies on other diseases have been carried out, such as acute kidney injury [3], Alzheimer's disease [4], and pulmonary arterial hypertension [5], and important progress has been made, and disease-related differentially expressed genes have been obtained.

The purpose of the present study was to explore the hub genes related to sepsis, construct protein interaction network, and find out key molecular targets. We downloaded two microarray datasets including GSE9692 and GSE95233 to screen the differentially expressed genes (DEGs) related to sepsis. Subsequently, the online tool DAVID was used for Gene Ontology (GO) analysis and Kyoto Encyclopedia of Genes and Genomes (KEGG) pathway enrichment analysis to explore the molecular functions and pathways related to sepsis, and finally protein-protein interaction (PPI) network analyses were conducted to elucidate the molecular mechanism of sepsis.

## 2. Material and Methods

### 2.1. Data Sources

The two datasets (GSE9692 and GSE95233) were selected and downloaded from the Gene Expression Omnibus (GEO) (https://www.ncbi.nlm.nih.gov/geo/) for the present study. Firstly, we used sepsis as the keyword for retrieval, and then, we selected *Homo sapiens* as the species information. Datasets containing more than 25 patients were selected. Patients with sepsis were divided into the “patient” group, while healthy people were divided into the “control” group. The platform used for both expression profiling arrays was GPL570 (HG-U133_Plus_2) Affymetrix Human Genome U133 Plus 2.0 Array. The dataset GSE9692 contained 29 children with sepsis septic shock and 16 healthy children, while the dataset GSE95233 included 102 septic subjects and 22 healthy volunteers. Ethical approval was not required for this study because we used public data for bioinformatics analysis.

### 2.2. Identification of DEGs

The DEGs were identified using the online tool GEO2R. The screening criteria for DEGs were adjusted *P* value <0.05 and |log fold change (LogFC) >2.0. Volcano plots were generated by Bioconductor (http://bioconductor.org/biocLite.R). The top ten and last ten DEGs sorted according to LogFC value were used for the heat map.

### 2.3. Functional and Pathway Enrichment Analyses

GO analysis was applied to conduct functional enrichment analysis, while KEGG analysis was adopted to cluster the possible pathways of these genes involving in. The DEGs screened in the previous step were used for GO analyses, KEGG pathway enrichment analyses, and PPI network analysis. The online tool DAVID (https://david.ncifcrf.gov/tools.jsp) was used for GO and KEGG analyses, and data visualization was completed by the R software.

### 2.4. PPI Network Construction and Hub Gene Identifcation

Search Tool for the Retrieval of Interacting Genes (STRING, https://string-db.org/) was applied to analyze protein interactions which were encoded by the filtered DEGs. The Cytoscape software was applied to show interaction results with a minimum combined score of 0.4. The plug-in component Molecular Complex Detection (MCODE) of Cytoscape was used to screen out the hub genes in the PPI networks.

## 3. Results

### 3.1. Identification of DEGs

The datasets GSE9692 and GSE95233 were selected and downloaded from GEO and were analyzed by GEO2R online tool. Then, the volcano plots of DEGs were generated, as shown in Figure 1. Total of 286 DEGs in GSE9692 were found in patients when compared with the controls, including 217 upregulated DEGs and 69 downregulated DEGs (Figure 1(a)), while there were 357 DEGs in GSE95233 (236 upregulated DEGs and 121 downregulated DEGs, Figure 1(b)). The heatmap plots of the top 10 upregulated genes and the top 10 downregulated genes were shown in Figures 2(a) and 2(b).

### 3.2. GO Annotation Analyses of DEGs

In order to screen out hub genes related to sepsis, David online analysis was applied to annotate the gene function. GO annotation analysis of GSE9692 indicated the differential genes participated in inflammatory responses, including regulation of immune effector process, regulation of leukocyte-mediated immunity, regulation of lymphocyte-mediated immunity, positive regulation of cytokine production, immune response-regulating signaling pathway, regulation of leukocyte-mediated cytotoxicity, and immune response-regulating cell surface receptor signaling pathway (Figure 3(a)). GO analysis of GSE95233 suggested DEGs involved in biological functions, such as T cell activation, leukocyte cell-cell adhesion, positive regulation of leukocyte activation, positive regulation of leukocyte cell-cell adhesion, and leukocyte-mediated immunity (Figure 3(b)). A total of 98 codifferentially expressed genes (co-DEGs) were obtained after the intersection of DEGs in the two datasets. GO analysis showed these 98 co-DEGs involved in biological functions, such as leukocyte-mediated immunity, regulation of cytokine production, regulation of immune effector process, regulation of lymphocyte-mediated immunity, defense response to fungus, and lymphocyte-mediated immunity (Figure 3(c)).

### 3.3. KEGG Pathway Enrichment Analyses of DEGs

By analyzing the signal pathway of DEGs, we can understand the significantly changed metabolic pathway in the state of disease, which is important for exploring the pathogenesis of disease. KEGG pathway analysis was conducted to identify the signal pathways of DEGs. KEGG pathway analysis suggested that the DEGs of GSE9692 associated with sepsis were related to different infections such as *Staphylococcus aureus* infection, malaria, leishmaniasis, legionellosis, influenza A, inflammatory bowel disease (IBD), amoebiasis, and immune response-related pathway (Figure 4(a)). KEGG pathway analysis of GSE95233 suggested that the DEGs were related to different infections such as tuberculosis, toxoplasmosis, *Staphylococcus aureus* infection, leishmaniasis, influenza A, IBD, HTLV-l infection, Epstein–Barr virus infection, and immune system diseases such as rheumatoid arthritis, primary immunodeficiency, and autoimmune thyroid disease (Figure 4(b)). KEGG pathway analysis showed that the intersecting DEGs were related to different infections such as *Staphylococcus aureus* infection, malaria, leishmaniasis, IBD, and amoebiasis (Figure 4(c)).

### 3.4. PPI Network and Hub Genes

In order to better understand the molecular mechanism of sepsis, we uploaded DEGs to STRING (https://string-db.org/) for PPI analysis, and then, visualized the importance of the relationship between proteins using the Cytoscape software. We submitted 200 genes of GSE9692, 241 genes of GSE95233, and 98 co-DEGs to STRING for PPI analysis, respectively, and identified some hub genes, such as IL-2-inducible tyrosine kinase (ITK), CD247, matrix metallopeptidase 9 (MMP9), CD3D, matrix metallopeptidase 8 (MMP8), killer cell lectin-like receptor subfamily K (KLRK1), and granzyme K (GZMK) (Figure 5).

## 4. Discussion

With the advent of the era of big data, bioinformatics is widely used in the research of various diseases, including sepsis. Although the survival rate of sepsis patients is increasing, the mortality rate is still 30–40% [2]. At present, the treatment of sepsis mainly includes anti-infection, fluid resuscitation, multiorgan function maintenance, and other comprehensive treatments [6, 7]. However, even with advanced support technologies such as extracorporeal membrane oxygenation (ECMO), the prognosis of sepsis is still poor [8]. High throughput microarray technology provides us with the possibility to understand the molecular mechanism of sepsis.

In this study, we performed bioinformatics analysis on two sepsis microarray datasets (GSE9692 and GSE95233) to screen a series of differentially expressed genes related to sepsis. We further analyzed the selected DEGs' signal pathway enrichment and gene annotation, and the results showed that DEGs associated with sepsis involved in inflammatory responses such as T cell activation, leukocyte cell-cell adhesion, leukocyte-mediated immunity, regulation of cytokine production, regulation of immune effector process, regulation of lymphocyte-mediated immunity, defense response to fungus, and lymphocyte-mediated immunity. KEGG pathway enrichment analysis showed that sepsis was related to bacterial and viral infections. Current research suggests that sepsis is a competition between pathogens and host immune system. The balance between proinflammatory system and anti-inflammatory system determines the disease trend of patients. Functional failure of T cell, B cell, DCs, and KCs usually occur in patients died of sepsis. Monocyte macrophage system is the inherent immune system of human body and plays an important role in the occurrence and development of sepsis [9].

Subsequently, the differentially expressed genes were analyzed by PPI to better understand the molecular mechanism of sepsis. Through PPI network analysis, we screened the most important hub genes, including ITK, CD247, MMP9, CD3D, MMP8, KLRK1, and GZMK.

ITK is a member of the TEC kinase family and the most important Tec kinase in T cells. Many studies have shown that ITK plays a critical role in the development and differentiation of T cells, promotes Th2, Th9, and Th17 responses, and then inhibits the expression of proinflammatory cytokines. Studies have shown that ITK is a key regulator of T lymphocytes and plays a critical role in the pathogenesis of autoimmune diseases [10, 11]. Inhibition of ITK by inhibitors has a certain beneficial effect on asthma, inflammatory bowel disease, and rheumatoid arthritis [12]. Studies have shown that ITK regulated thermal homeostasis in sepsis through affecting mast cells [13].

CD247 is located in band 2 of region 24 of the long arm of chromosome 1 and belongs to the CD3Z/FCERIG family, with a length of 88 kb. CD247 is a main factor leading to linking antigen recognition and intracellular signal transduction of T lymphocytes. The coding product of CD247 gene is CD3/T-cell receptor complex (CD3/TCR complex), which is a complex formed by the noncovalent binding of T cell antigen receptor and CD3 molecule [14]. It is the main unit of T cell recognition antigen and signal transduction. Interestingly, previous studies have shown that CD3D encodes the *δ* subunit of transmembrane CD3 antigen complex [15]. The main function of TCR is to recognize and bind the MHC antigen peptide complex, while CD3 further transfers the signal recognized by TCR into T lymphocytes to induce T lymphocyte activation, and the TCR/CD3 membrane expression level determines the initiation of T lymphocyte activation. Studies have shown that the gene CD247 is also involved in other autoimmune diseases, such as systemic lupus erythematosus [16, 17], rheumatoid arthritis [18], and systemic sclerosis [19], which shows that CD247 is closely related to the occurrence of autoimmune diseases. The expression of CD247 can affect the development of T cells and lead to abnormal activation of T lymphocytes. The low expression of CD247 can cause damage to the immune system and affect lymphocyte proliferation and cytokine production. The expression of CD247 is gradually downregulated during the development from sepsis to septic shock [20]. Jiang et al. found that CD247 was the hub gene of sepsis through bioinformatics analysis [21].

Studies have shown that MMP9 is associated with inflammation and inhibits platelet aggregation [22]. Previous studies have proved that MMP9 is upregulated in sepsis patients compared with healthy people, and MMP9 expression can be used as a prognostic biomarker of sepsis. In addition, MMP9 has high accuracy in the diagnosis of sepsis, and the result of ROC curve analyses showed the area under the curve of MMP9 was 0.967, indicating that MMP9 plays an important role in the pathogenesis of sepsis.

Viral or bacterial infection can lead to the induction of KLRK1 ligands on cells to activate the immune system to recognize and eliminate them [23]. Studies have reported that CD3D is actually involved in the activation of T lymphocyte immune-related pathways, and the lack of CD3D may lead to the damage of immunity [24]. GZMK is mainly expressed in T lymphocytes and can also promote the release of proinflammatory cytokines, TNF-*α*, IL-1, IL-6, and MCP-1 [25]. Almansa et al. evaluated gene expression profiles in patients with sepsis and found the extent of organ failure and mortality in sepsis was associated with MMP8, CD3D, and KLRK1 [26].

In conclusion, the present study revealed an unbalanced immune response at the transcriptome level of sepsis and identified genes for potential biomarkers of sepsis, such as ITK, CD247, MMP9, CD3D, MMP8, KLRK1, and GZMK.

## Figures and Tables

**Figure 1:** Volcano plots of differentially expressed genes (DEGs) in GSE9692 and GSE95233. (a, b) The volcano plots of DEGs in GSE9692 and GSE95233, respectively.

**Figure 2:** The heatmap plots of the top 10 upregulated genes and the top 10 downregulated genes. (a) GSE9692. (b) GSE95233.

**Figure 3:** Gene Ontology (GO) analyses of DEGs. (a) GO analysis of DEGs of GSE9692. (b) GO analysis of DEGs of GSE95233. (c) GO analysis of co-DEGs of GSE9692 and GSE95233.

**Figure 4:** Kyoto Encyclopedia of Genes and Genomes (KEGG) analyses of DEGs. (a) KEGG analysis of DEGs of GSE9692. (b) KEGG analysis of DEGs of GSE95233. (c) KEGG analysis of co-DEGs of GSE9692 and GSE95233.

**Figure 5:** The protein-protein interaction (PPI) networks based on the screened differentially expressed genes (DEGs). (a, b, c) The PPI networks based on screened DEGs of GSE9692. (d, e, f) The PPI networks based on screened DEGs of GSE9692. (g, h, i) The PPI networks based on screened co-DEGs of GSE9692 and GSE95233.

## Data Availability

The data used to support the findings of this study are available from the corresponding author upon reasonable request.
